The article "Synthesis, Characterization, and Antiproliferative Effect of CuO-TiO2-Chitosan-Amygdalin Nanocomposites in Human Leukemic MOLT4 Cells" was published in 2022. Journal: Bioinorg Chem Appl.

# Synthesis, Characterization, and Antiproliferative Effect of CuO-TiO_2_-Chitosan-Amygdalin Nanocomposites in Human Leukemic MOLT4 Cells

**DOI:** 10.1155/2022/1473922

**Published:** 2022-09-26

**Authors:** Abozer Y. Elderdery, Badr Alzahrani, Siddiqa M. A. Hamza, Gomaa Mostafa-Hedeab, Pooi Ling Mok, Suresh Kumar Subbiah

**Affiliations:** ^1^Department of Clinical Laboratory Sciences, College of Applied Medical Sciences, Jouf University, Sakaka, Saudi Arabia; ^2^Faculty of Medicine, Department of Pathology, Umm Alqura University Algunfuda, Mecca, Saudi Arabia; ^3^Pharmacology & Therapeutic Department, Medical College, Jouf University, Sakaka, Saudi Arabia; ^4^Department of Biomedical Sciences, Faculty of Medicine & Health Sciences, Universiti Putra Malaysia, 43400 UPM Serdang, Seri Kembangan, Selangor, Malaysia; ^5^Centre for Materials Engineering and Regenerative Medicine, Bharath Institute of Higher Education and Research, Chennai, India

## Abstract

The main aim of this study was to synthesize copper oxide- (CuO-) titanium oxide- (TiO_2_-) chitosan-amygdalin nanocomposites (CTCANc) and to characterize them physically and biologically (antimicrobial and anticancer activity using MOLT4 blood cancer cell line) to endorse their useful applications as potential drug candidates in anticancer avenues. CuO-TiO_2_-chitosan-amygdalin nanocomposites were synthesized according to standard, reported methods. Physical characterization of the nanocomposites was performed using methods like X-ray diffractometer (XRD), and morphological and ultrastructural analysis of nanocomposites were done using electron microscope scanning and transmission. FTIR was recorded using a Perkin-Elmer spectrometer, and photoluminescence (PL) spectra were done using the spectrometer. Further, antibacterial activities were assessed using standard bacterial cultures. To demonstrate the nanocomposite's anticancer effects, MTT assay, morphological analysis, apoptosis studies using acridine orange/ethidium bromide (AO/EtBr) dual staining, reactive oxygen species (ROS) analysis, and levels of antioxidant enzymes were analyzed using the MOLT4 blood cancer cell line. Synthesized nanocomposites were characterized using XRD and showed various peaks, respectively, for CuO-TiO_2_, amygdalin, and chitosan. MTT assay indicated an IC_50_ value of 38.41 *μ*g/ml concentration of CTCANc. Hence, 30 and 40 *μ*g/ml were used for the subsequent experiments. Morphological analysis, staining for apoptosis using AO/EtBr, mitochondrial membrane potential (MMP or ΔΨm) analysis, ROS analysis, and determination of the SOD, CAT, MDA, and GSH levels were performed. Observations like a significant loss of morphology, induction of apoptosis, elevated ROS, and decreased MMP were significant in 30 and 40 *μ*g/ml nanocomposite-treated cells when compared to control cells. The bimetallic nanocomposites exhibited typical nanocomposites characteristics and significant antibacterial and anticancer effects. The study results endorse the antibacterial, anticancer activity of CuO-TiO_2_-chitosan-amygdalin nanocomposites and strongly suggest that further in-depth research using CuO-TiO_2_-chitosan-amygdalin nanocomposites could reveal their efficacy in the clinical scenario.

## 1. Introduction

Applications of metal oxides in the form of bimetallic nanosized metal oxides, like copper oxide (CuO) and titanium oxide (TiO_2_), have gained broad scope applications in catalysis, biomedical research, drug development, and engineering applications like solar cells [1, 2]. Chemically, CuO and TiO_2_ were characterized as semiconductors with photoconductive and photochemical properties [3]. Notably, CuO and TiO_2_ were well-appreciated agents in the areas of nanocomposite developments due to their innate nature to combine in desirable ways with unique physicochemical properties [4]. There are several key points mentioned in the earlier reports: highly stable, nontoxic, readily available, and possessing a narrow band gap, with special emphasis on the use of CuO and TiO_2_. Hence, CuO and TiO_2_ bimetallic nanocomposites have gained wide interest for researchers in an array of fields, including drug development [5–7].

Polycationic chitosan, biologically prevalent, is nontoxic and biodegradable, with multiple, interesting properties [8]. As an edible coating and packaging material, chitosan is utilized widely in the food and pharmaceutical industry. Through photocatalysis, it can be used for the treatment of wastewater in addition to having an adsorbent capacity [9]. In addition to healing wounds and wound regeneration, chitosan is antimicrobial, antioxidant, anticancer, and immunomodulatory, making it a suitable candidate for targeted therapy [10–12].

In the recent decade, nanocomposites derived from plant-based bioactive components have gained significant attention for their utility in various human drug development avenues, for example, the development of using Laetrile, a phytochemical present in beans, sorghum, clover, and rosacea plants like apple, peach, lima, plum, bayberry, and seeds of almonds [13]. Amygdalin is an aromatic cyanogenic compound that is widely used in countries of Asia and Europe. The seeds of *Prunus* species contain amygdalin, also known as vitamin B17, which is traditionally used to treat leprosy, leukoderma, bronchitis, and other minor ailments.

Recent *in vivo* and *in vitro* studies, however, have validated the compound's pharmacological activities, including anti-inflammatory, antitumor, antiatherosclerosis, antifibrotic, immunomodulatory, analgesic, and an agent that improves digestive and reproductive system functions, alleviates neurodegeneration, and lowers blood glucose levels [13–15]. Amygdalin is also widely recommended for cancer phytotherapy against breast, lung, bladder, prostate, cervical, and renal cancers [16] and also mediates effect on regulating immune functions [17], in addition to its potentiality as an anticancer, antidiabetic agent [18] and its utility in the treatment of neurological disorders [13] and lung disorders [16, 17] in recent periods. Amygdalin increases polyhydroxyalkanoates(PHA)-induced production of peripheral blood lymphocytes and promotes the production of interleukin-2 and interferon-*γ* to inhibit transforming growth factor-*β*1 secretion by stimulated peripheral blood lymphocytes [19]. Although high doses of amygdalin (due to its enzymatic degradation) have been associated with cyanide poisoning in various anticancer studies, research studies are continuously pursued to determine its optimum usage and its mechanisms of action *in vitro* [9].

Amygdalin can induce apoptosis in a variety of cancer cells by increasing proapoptotic Bax expression and decreasing antiapoptotic Bcl-2 expression [20]. Despite the understanding that amygdalin primarily affects anticancer effects by its antiapoptotic effect, many reports denote that amygdalin mediates various biological functions and the precise mechanisms by which it induces apoptotic effects at the cellular level remain unknown. Hence, the need for research studies aiming to understand its anticancer functions in various cancer models is greatly warranted [21, 22].

Based on such literature, the present study aims to generate a hybrid nanocomposite from amygdalin and chitosan conjugated with metal ions and demonstrate their anticancer properties against the human leukemic MOLT4 cell line. As a result, we developed a bimetallic nanocomposite to demonstrate the anticancer properties of amygdalin by conjugating it with bimetallic oxides. In the *in vitro* study using MOLT4 blood cancer cells, we demonstrated significant antioxidant, antimicrobial, and anticancer effects of plant-derived amygdalin-copper oxide-titanium oxide-chitosan nanocomposites (CTCANc).

## 2. Methodology

### 2.1. Chemicals

Titanium oxide, acridine orange, MTT, rhodamine 123, amygdalin, copper II nitrate hexahydrate ethidium bromide, and antibiotic penicillin-streptomycin were purchased from Sigma-Aldrich chemical company (Merck & Co., Inc. USA). Gibco Dulbecco's Modified Eagle (DMEM) Medium and Fetal Bovine Serum (FBS) were obtained from Thermo Scientific, USA. We purchased a ROS detection kit from Nanjing KeyGen Biotech Co., Ltd.

### 2.2. Nanocomposites of CuO-TiO_2_-Chitosan-Amygdalin Synthesized

CTCANc were synthesized by mixing 500 mg of TiO_2_ nanoparticles with 0.1 M copper (II) nitrate hexahydrate and dissolved in 1% acetic acid in 50 mL of water. The CuO-TiO_2_-chitosan solution was also mixed with 50 mg of phytocomponents of amygdalin. A solution of CuO-TiO_2_-chitosan-amygdalin was then added drop by drop with 0.1 M NaOH solution. The residual dark-colored substances were heated at 37°C for 3 hours. At various stages, ethanol and deionized water solutions were used to clean the nanopowder using a centrifuge at 15,000 rpm for 40 minutes at −3°C. We dried the black residue at 120°C for 2 hours and calcined it at 600°C for 5 hours.

### 2.3. CuO-TiO_2_-Chitosan-Amygdalin Nanocomposites Characterized

X-ray diffractometer (XRD) (model: X'PERT PRO PANalytical) analysis was performed on CuO-TiO_2_-chitosan-amygdalin nanocomposites samples. A monochromatic CuK*α* diffraction beam of wavelength 1.5406 Å was used to measure the diffraction patterns for CuO-TiO_2_-chitosan-amygdalin nanocomposites in the 2*θ* range between 25° and 80°. An Energy Dispersive X-ray Spectrometry (EDX) microscope (Carl Zeiss Ultra 55 FESEM, model: Inca) was used for the examination of the CuO-TiO_2_-chitosan-amygdalin nanocomposites. TEM (Tecnai F20 model) was used to examine the morphologies of the CuO-TiO_2_-chitosan-amygdalin nanocomposites. A Perkin-Elmer spectrometer was used to record FTIR data in the range of 400–4000 cm^−1^. A Lambda 35 spectrometer was used to study the absorption spectra of CuO-TiO_2_-chitosan-amygdalin nanocomposites between 200 and 1100 nm. Perkin-Elmer-LS spectrometer was used to take photoluminescence (PL) spectra.

### 2.4. Nanocomposites Containing CuO-TiO_2_-Chitosan-Amygdalin Have Antibacterial Properties

The antibacterial activity of target microorganisms was studied using an agar-based well diffusion method that included Gram-positive (*S. aureus* and *S. pneumonia*) and Gram-negative (*K. pneumonia* and *E. coli*) strains. Petri discs were spread with separate bacterial pathogens on sterile nutrient agar, and 25 mL of sterile nutrient agar was poured into a sterile Petri plate. In a 5% sterilized dimethyl sulphoxide solution, CuO-TiO_2_-chitosan-amygdalin nanocomposites were dissolved at concentrations of 1, 1.5, and 2 mg/mL. Zones of inhibition were also evaluated after 24 hours on Petri plates incubated overnight at 37°C. A common antibiotic, amoxicillin (30 g/ml), was used as a positive control, and triplicate assays were performed.

### 2.5. Cell Culture

The ATCC in the United States provided us with human MOLT4 cells, which were cultured in 10% FBS and Eagle's Minimum Essential Medium with 1% penicillin-streptomycin. After 48 hours of incubation at 37°C with 5% CO_2_, cells were subcultured with 0.25 percent trypsin-EDTA solution at 80% confluency.

### 2.6. Viability Assay Using MTT

A 96-well clear bottom MTT plate was used to assess the cytotoxicity of amygdalin bimetallic nanocomposites to MOLT4 cells. A variety of doses (10, 20, 30, 40, 50, and 60 *μ*g/ml) of amygdalin bimetallic nanocomposites were applied to MOLT4 cells for 24 hours after seeding into 96-well plates. Following the treatment period, cells were washed with sterile 1 X PBS at room temperature (RT) using centrifugation (1,000 × *g*, 4°C for 5 min), and 20 *μ*l of MTT (0.5 mg/ml) was added to each well and incubated in the dark for 4 hours, with regular monitoring under an inverted microscope for the formation of blue-colored formazan crystals. Following the production of formazan crystals, the media from each well were gently removed by centrifugation, and 150 *μ*l of dimethyl sulphoxide (DMSO) was added to digest the crystals before being agitated on an orbital shaker to obtain a homogeneous solution. The optical density was determined using a Multiskan FC microplate reader (Thermo Fisher Scientific, USA) at 570 nm [23].

MOLT4 cells were grown in 12-well plates at a density of 1.5 × 10^5^ cells/well for 24 hours before being treated with nanocomposites (IC_50_ values of 30 and 40 *μ*g/ml) for 24 hours. After treatment with nanocomposites, MOLT4 cells were washed with cell culture grade 1X PBS and centrifuged (1,000 × *g*, 4°C for 5 minutes). After gentle washing, MOLT4 cells were immobilized for 10 minutes at room temperature with 4 percent paraformaldehyde (Sigma-Aldrich) in 1 X PBS (RT). An inverted phase-contrast microscope (IX73; Olympus Corporation, Tokyo, Japan) was used to detect morphological changes, and experiments were performed in triplicate.

### 2.7. Analysis of Cell Morphology to Detect Apoptotic Cell Death

MOLT4 cells (2 × 10^6^ cells/well) were seeded into sterile 6-well plate dishes for 24 hours before being treated with amygdalin bimetallic nanocomposites with IC_50_ concentrations (30 and 40 *μ*g/ml). Following the treatment protocol, MOLT4 cells were treated with 1 M of AO/EtBr at 37°C for 5 minutes in the dark. Finally, the stained cells were photographed and viewed using a fluorescence microscope's green and red channels (20X) (ZOE Cell Imager, BioRad, USA). The fluorescence intensity of AO/EtBr was measured in triplicate using a SpectraMax M2 Multimode Microplate Reader (Molecular Devices, USA).

Using rhodamine 123 dye, we investigated the permeability of mitochondrial membranes in nanocomposites-treated and untreated cells. The nanocomposites were applied to 6-well plates containing MOLT4 (2 × 10^6^ cells/well) cells and incubated for 24 hours at 37°C. After being rinsed twice in PBS, the cells were stained with 1 mM rhodamine 123 for 30 minutes before being incubated in the dark for 15 minutes. Images of fluorescent cells were produced after examining the dyed cells (20X) with a fluorescence microscope (ZOE Cell Imager, BioRad, USA). Three independent experiments were carried out to assess the intensity of Rh123 fluorescence using a SpectraMax M2 Multimode Microplate Reader (Molecular Devices, USA).

### 2.8. ROS Production Detection Assay

The analysis and quantification of ROS were done with minor modifications based on the work of Huang et al. [24]. MOLT4 (2 × 10^6^ cells/well) cells were treated for 24 hours with two different doses (30 and 40 *μ*g/ml) of nanocomposites. Following the treatment protocol, MOLT4 cells were washed with sterile PBS and resuspended in serum-free culture media with 10 *μ*M dichloro-dihydro-fluorescein diacetate (DCFH-DA). The cells were treated for 10 minutes with hydrogen peroxide (H_2_O_2_) (50 g/ml) as a positive control. Finally, ROS were imaged using fluorescence microscopy (ZOE Cell Imager, BioRad, USA) with DCFH-DA excitation and emission wavelengths. The intensity of the DCFH-DA fluorescence was measured using a SpectraMax M2 Multimode Microplate Reader (Molecular Devices).

### 2.9. Evaluation of SOD, CAT, GSH, and MDA Intracellular Activities

MOLT4 cells (2 × 10^6^ cells/well) were grown and treated with nanocomposites (30 and 40 *μ*g/ml). After the cells have been exposed, they were extracted, washed twice with PBS, lysed in cell lysis buffer, and centrifuged at 12,000 × *g* for 10 minutes at 4°C, and the supernatant was collected. The quantities of SOD, CAT, MDA, and GSH in cell lysates were measured using the BCA technique, as directed by the manufacturer. SOD activity was measured using hypoxanthine and xanthine oxidase methods [25]. The rate constant of H_2_O_2_ decomposition was used to calculate catalase activity as U/mg protein [26]. Thiobarbituric acid was employed to assess lipid peroxidation [27], and MDA levels were expressed in nanomoles per milligramme of protein. GSH concentration in whole cells was determined using an enzymatic recycling approach including glutathione reductase and 5-dithio-5′, 5′-dinitrobenzoic acid (DTNB), in which DTNB oxidized GSH and NADPH oxidized it, and GSH was expressed as nmol/mg protein [27].

### 2.10. Statistical Analysis

The average of three separate experiments was derived in this study by combining the mean and standard deviation. To examine statistical significance, we utilized GraphPad Prism version 5, and the *p* value of <0.05 was used to determine statistical significance.

## 3. Results

### 3.1. Characterization Analysis of CuO-TiO_2_-Chitosan-Amygdalin Nanocomposites

Figure 1(a) depicts X-ray diffraction patterns of nanocomposites produced. XRD patterns show 2θ (angle values) for chitosan at 10.57° and 19.08°, CuO peaks at 32.36°, 35.59°, 38.71°, 58.23°, 61.55°, and 66.11°: JCPDS Card (005-0661) [28], TiO_2_ peaks at 24.27°, 25.10°, 37.66°, 48.16°, 53.96°, and 56.14°. In DLS, the spectrum of nanocomposites was found at 137 nm (Figure 1(b)). As a result of hydrodynamic size, the nanocomposites exhibit increased particle size in DLS when compared to TEM and XRD.

The surface morphology of synthesized nanocomposites was identified by FESEM/TEM/image, as illustrated in Figure 2. The nanocomposites have a spherical structure with an average particle size of 45 nm, which is consistent with the XRD data. The creation of the CuO monoclinic structure in the TiO_2_-chitosan-amygdalin matrix was confirmed by the selected area of the electron diffraction (SAED) pattern (Figure 3). The EDAX spectrum of the nanocomposites is shown in Figure 2(b), with the atomic percentages found to be 12.04% (C), 7.54% (N), 16.61% (Zn), 12.58% (Ti), and 51.23% (O).

FTIR spectrum of synthesized nanocomposites is depicted in Figure 4(a). It can be observed that, along with the broad range of OH and NH peaks by hydrogen bonds and the amide I group, the typical chitosan characteristics peaks are observed at 3427 and 1647 cm^−1^ (C-O stretching along with the N-H deformation mode) [29]. Meanwhile, the amygdalin properties reached a peak: -C-H(CH_2_) peaks at 2924 and 2856 cm^−1^, C-O stretching vibration observed at 1113 cm^−1^, and -HC=CH out of plane bending observed at 958 cm^−1^, respectively. In addition, the stretching vibration of the Ti-O and Cu-O bonds also appeared at around 710 cm^−1^ and 532 cm^−1^ [30]. Thus, the FTIR results demonstrate the formation of the nanocomposite.

UV-visible spectroscopy was used to measure the pattern of nanocomposites, which revealed an absorbance peak edge at 395 nm (Figure 4(b)), which was the same as others' reported value for CuO NPs of 383 nm [31]. The PL spectra of nanocomposites with an excitation wavelength of 325 nm at room temperature are shown in Figure 4(c). The emission values of the produced nanocomposites are observed at 363 nm, 422 nm, 441 nm, 488 nm, and 520 nm. The recombination of electrons in the conduction band and holes in the valence band is responsible for the NBE emissions (UV) observed at 363 nm. The deep emission of oxygen vacancies, Cu interstitials, and Ti interstitials resulted in three blue emissions at 422 nm, 441 nm, and 488 nm. The 520 nm (green emission) is caused by recombining a photo-generated hole with a single ionized electron in valence band nanocomposites.

### 3.2. Antimicrobial Activity of Nanocomposites

Using the well diffusion method, the antibacterial activity of nanocomposites was tested again for Gram-positive (*S. aureus* and *S. pneumonia*) and Gram-negative (*K. pneumonia* and *E. coli*) bacterial strains (Figure 5(a)). According to the research, nanocomposites can kill bacteria based on their concentration, and increasing concentration enhances antibacterial activity (zone of inhibition). As demonstrated in Figure 5(b), nanocomposites are more effective than conventional antibiotic amoxicillin.

### 3.3. CuO-TiO_2_-Chitosan-Amygdalin Nanocomposites Exhibit Anticancer Potential

#### 3.3.1. MTT Test for Determining Cell Viability

An MTT assay was used to assess the cytotoxicity of nanocomposites on the MOLT4 cell line, and the results showed that the IC_50_ concentration for nanocomposites was 38.41 *μg*/ml for MOLT4 cells. Anticancer experiments were conducted for 24 hours at 30 and 40 *μg*/ml concentrations based on the IC_50_ value (Figure 6(a)). MOLT4 cells were treated for 24 hours with nanocomposites at doses of 30 and 40 *μg*/ml. An inverted light microscope was used to examine the cells, and the nanocomposites-treated cells showed significant (*p* < 0.05) morphological changes when compared to the control untreated cells (Figure 6(b)).

#### 3.3.2. MOLT4 Morphological Characterization during Apoptosis Using Fluorescent Staining

MOLT4 cells were fixed, stained with acridine orange and ethidium bromide, and observed using a fluorescence microscope after being treated with nanocomposites at 30 and 40 *μ*g/ml concentrations for 24 hours. When compared to control cells, nanocomposites-treated cells had a considerably (*p* < 0.05) higher number of apoptotic cells (Figure 7).

#### 3.3.3. The Mitochondrial Membrane Potential (ΔΨm) in Nanocomposite-Treated MOLT4 Cells Was Determined

During oxidative phosphorylation, mitochondrial membrane potential (ΔΨm) is essential for energy storage. Rh123 staining was used to determine the levels of MMP in the nanocomposite (30 or 40 *μ*g/ml)-treated MOLT4 cells. As presented in Figure 8, a bright green fluorescence was detected in the control cells, indicating a higher MMP level. However, the nanocomposites-treated cells exhibited a lower green fluorescence signal, suggesting decreased MMP activity.

#### 3.3.4. ROS Levels in MOLT4 Cells Were Increased by CuO-TiO_2_-Chitosan-Amygdalin Nanocomposites

MOLT4 cells were cultivated overnight before being treated with nanocomposites (30 and 40 *μ*g/ml) for 24 hours in the dark. There was an increase in ROS creation in nanocomposites-treated cells, but there was little or no ROS formation in MOLT4 control cells (Figure 9).

#### 3.3.5. Nanocomposites of CuO-TiO_2_-Chitosan-Amygdalin Produced Oxidative Stress

The impact of CuO-TiO_2_-chitosan-amygdalin nanocomposites on cellular oxidative stress was also investigated by measuring antioxidant enzyme levels such as SOD, CAT, GSH, and MDA. CuO-TiO_2_-chitosan-amygdalin nanocomposites in concentrations of 30 and 40 *μ*g/ml decreased SOD, CAT, and GSH levels while increasing MDA levels (Figure 10).

## 4. Discussion

The need for better anticancer agents with less or minimal side effects with higher efficacy has been of the utmost need in recent decades. Tyrosine kinase inhibitors (TKIs) are commonly effective at managing CML for long periods, and Imatinib (Gleevec®), Dasatinib (Sprycel®), Nilotinib (Tasigna®), and Bosulif (Bosulif®) are the three TKIs approved for primary therapy for chronic phase CML. When these do not work, chemotherapy may be combined with targeted drug therapy [32]. CML was most effectively treated with synthetic interferon, i.e., interferon-alpha before tyrosine kinase inhibitors became available [33]. When chemotherapy or interferons are not effective against CML, TKIs are the most common form of treatment other than stem cell transplantation. Additionally, if leukemia spreads to the spleen, a splenectomy may be necessary [34].

In such a context, the role of natural plant-based agents in discovering their latent potential in cancer phytotherapy has always been in the spotlight, and lately, the development of bimetallic nanocomposites employing plant-based phytochemicals has received great relevance. Plant-derived phytochemicals combined with metal oxides in the form of nanocomposites were discovered to have higher efficacy in anticancer and other clinical medication development pathways [35, 36]. Here, we have synthesized and characterized the nanocomposites. Amygdalin nanocomposites were then scrutinized to find their ability as an antimicrobial and anticancer agent against the *in vitro* MOLT4 blood cancer cell line.

Synthesized nanocomposites showed specific and unique patterns of nanocomposite material as observed from TEM, SEM, and XRD analysis. Our findings show that the steric effects and intermolecular hydrogen bonding between the CuO-TiO_2_-chitosan-amygdalin matrixes contribute to the creation of nanocomposites. The Debye–Scherrer formula calculated the average crystallite size of the CuO-TiO_2_-chitosan-amygdalin matrix to be 45 nm. These nanocomposites were also tested for antibacterial activity against *S. aureus*, *S. pneumonia*, *K. pneumonia*, and *E. coli* bacterial strains. Our findings revealed that the nanocomposites we developed were antimicrobially effective against pathogenic bacteria of both types, as determined by Gram stain. In addition, studies on the antimicrobial properties of amygdalin, which is found in crushed apple seeds, bitter almonds, and peaches extract, have revealed synergistic effects against a variety of pathogenic bacteria, including *E. coli*, *Staphylococcus aureus*, *Streptococcus pyogenes*, and *Pseudomonas aeruginosa* [37–39].

The antibacterial activity of these nanocomposites is influenced by several variables, including oxidative stress and the generation of free radicals (ROS), changes in particle size, surface-volume-ratio, an increase in oxygen vacancies (surface defects), electrostatic attraction, the ability of the reactant molecules (chitosan) to diffuse, and the release of Cu^2+^/Ti^4+^ ions [40]. Furthermore, the green emission visible at 520 nm in the PL spectrum is caused by a singly ionized oxygen vacancy, and surface defects in CuO-TiO_2_-chitosan-amygdalin, such as oxygen vacancies, are critical factors to confer biocidal effect. The surface defects, especially oxygen vacancies, cause more ROS to be generated in the cell cytoplasm through a water-splitting mechanism [41], leading to an active source of singlet oxygen and hydroxide radicals.

The ability of CuO-TiO_2_-chitosan-amygdalin nanocomposites can be attributed to their ability to induce ROS generation upon exposure to bacterial strains. Additionally, it could exert its effect by its ability to penetrate the cell membranes of bacterial strains and inhibit their growth mechanisms employing disorganization to their cell membranes [42]. Our results are in conjunction with previous reports and thereby denote that metal oxide nanoparticles are capable of inducing bacterial growth inhibition via ROS or by penetrating the membranes of bacterial cells [43–45].

The anticancer activity of these nanocomposites was subsequently investigated *in vitro* utilizing MOLT4 blood cancer cell lines. IC_50_ values between 30 and 40 *μ*g/ml (38.41 µg/mL) for the nanocomposites were determined using the MTT assay. Morphological analysis using the MOLT4 blood cancer cell line showed significant alterations in treated cells when compared with the control cells. The observed morphological changes can be attributed to the elevated ROS species generated in the cells upon exposure to CuO-TiO_2_-chitosan-amygdalin nanocomposites. Our results are in support of the earlier research findings that reveal that chitosan nanoparticles are capable of inducing ROS favoring cancer cell death [44].

Further, to check whether CuO-TiO_2_-chitosan-amygdalin nanocomposites mediate apoptotic induction, we have performed AO/EtBr staining in MOLT4 cells treated with nanocomposites. As expected, the treated MOLT4 blood cancer cell line showed significant staining for AO/EtBr, which denotes the loss of membrane integrity due to nanocomposite exposure. This ability of CuO-TiO_2_-chitosan-amygdalin nanocomposites to induce morphological changes could be the direct pathological effect of supraphysiological ROS and oxidative damage induced by these nanocomposites as stated earlier or via its ability to directly penetrate the cell membranes of MOLT4 cell line, thereby causing stress within cells [46].

In addition to the above, to confirm the ability of these nanocomposites to induce reactive oxygen species in a cell culture medium, we have performed the ROS analysis experiment using fluorescent dye DCFH-DA. Our results showed that nanocomposites exhibited induction of ROS in MOLT4 cells, which could be the reason for their ability to induce cytotoxicity, morphological changes, and oxidative stress as observed in our preliminary experiments. Earlier reports have also documented that engineered nanoparticles are capable of inducing ROS in biological systems [47], and our present results also support such findings. The ROS findings of this study strongly suggest that these nanocomposites due to their ability to induce ROS and oxidative stress, in conjunction with their ability to penetrate the cell membranes of MOLT4 cells, could lead to altered mitochondrial functions,therebyinducing activation of caspases.

Since MDA is one of the main products of lipid peroxidation, its concentration indicates the rate and intensity of lipid peroxidation within the cells. In our study, compared to control cells, CuO-TiO_2_-chitosan-amygdalin nanocomposites (30 and 40 *μ*g/ml) significantly elevated MDA levels (nmol/g) and significantly decreased GSH and CAT activities (*p* < 0.05). Furthermore, the findings of this study suggest that a decrease in MMP levels was accompanied by a decrease in dye accumulation in the mitochondria, which could be linked to the creation of a large number of reactive oxygen species (ROS). ROS induces apoptosis by depolarizing the mitochondrial membrane, which increases lipid peroxidation by-products (TBARS) and decreases antioxidant enzyme activity (SOD and CAT). By assessing endogenous antioxidant levels, these nanocomposites were examined for anticancer and antioxidant activities in MOLT4 cell lines, and the large concentration of reactive oxygen species that happens during carcinogenesis might play a significant role in oxidative damage. As a result, the antioxidant enzymes may increase or decrease. The activities of SOD and CAT were found to be higher in untreated MOLT4 cells (control) than in CuO-TiO_2_-chitosan-amygdalin nanocomposites-treated MOLT4 cell lines in this study. SOD and CAT activity were found to be higher in hepatoma (HepG-2) cell lines, as well [48].

The current study's TBARS and antioxidant enzyme findings are consistent with prior research on colon cancer cells [49] and Hela cells [50], and they also suggest that ROS formation by nanocomposites mediates the observed anticancer impact. These findings corroborated our current findings, which showed that SOD and CAT activity in MOLT4 cells were higher than in CuO-TiO_2_-chitosan-amygdalin nanocomposites-treated cell lines. GSH content was shown to be lower and TBARS content to be higher in nanocomposites treated with MOLT4 cell lines, while GSH levels were reported to be low in individuals with chronic alcoholic liver disease and liver cancer. Low GSH levels have been observed in tumor cells, which could be due to changes in the tumor cells' defense system [51, 52].

The modulated status of the antioxidants in the MOLT4 cells upon treatment with the CuO-TiO_2_-chitosan-amygdalin nanocomposites, in particular, the deterioration in the levels of SOD and CAT, indicates that both enzymes could predominantly be associated with the elimination of superoxide radicals and H_2_O_2_ accumulation. The study results thus highlight the potential anticancer activity of the nanocomposites. Since nucleus-targeting or nuclear membrane-penetrating nanocomposites could prove more beneficial to precision nanomedicine in humans' fight against blood cancer than membrane-specific ones, the present study synthesized, designed, and applied cellular nucleus-specific CuO-TiO_2_-chitosan-amygdalin nanocomposite for demonstrating its potential to alter subcellular organelle status and induce apoptosis.

## 5. Conclusion

Together, our results showed that CuO-TiO_2_-chitosan-amygdalin nanocomposites mediated significant antimicrobial and anticancer effects via generating ROS, oxidative stress, and inducing apoptosis. Further insight concerning the molecular mechanisms would enable and ascertain the utility of the CuO-TiO_2_-chitosan-amygdalin nanocomposites in cancer therapy.

## Figures and Tables

**Figure 1:** Morphology and particle size and of nanocomposites: (A) X-ray diffraction patterns of CTCANc (a). DLS measurement of size (b).

**Figure 2:** FESEM (a) and EDAX (b) images of nanocomposites.

**Figure 3:** TEM images (a-c) and SAED (d) pattern of nanocomposites.

**Figure 4:** FTIR (a), UV-Vis absorbance (b), and photoluminescence spectra (c) analysis of nanocomposites.

**Figure 5:** Antimicrobial effect of CuO-TiO_2_-chitosan-amygdalin nanocomposite. Bacterial strains tested in this investigation included Gram-positive and Gram-negative strains (a); *S aureus* (A), *S pneumonia* (B), *K pneumonia* (C), and *E coli* (D). CuO-TiO_2_-chitosan-amygdalin nanocomposites zone of inhibition quantitative measurements (b). Experiments were carried out in triplicate, values were expressed as mean ± SD, and typical photos are displayed here.

**Figure 6:** CTCANc exhibited cytotoxicity in MOLT4 cells. The viability of MOLT4 cells was determined using the MTT assay using various doses (10−60  *μ*g/ml) of nanocomposites, and the mean±SD of three independent experiments is reported (a). Representative images (20X) for the triplicate set of studies are shown (b).

**Figure 7:** Apoptotic effect of CTCANc in the blood cancer MOLT4 cells. We used AO and EtBr (1 : 1) to color control and treated cells with nanocomposites (30 and 40*μg*/ml, 24 hr), and statistical significance was calculated as ^*∗*^*p* < 0.05 and ^#^*p* < 0.001 based on a comparison with “control.”

**Figure 8:** In the MOLT4 cell line, CTCANc produced intracellular ROS. The oxidative stress caused by nanocomposites was stained with DCFH-DA.

**Figure 9:** MOLT4 cell line mitochondrial membrane potential was affected by CTCANc. These fluorescence images showed a decreased mitochondrial membrane permeability after exposure to CuO-TiO_2_-chitosan-amygdalin nanocomposites.

**Figure 10:** Antioxidant enzymes SOD, CAT, GSH, and MDA were persuaded by CTCANc in MOLT4 cell line. Active MDA (a), CAT (b), SOD (c), and GSH (d) levels were measured colorimetrically in the MOLT4 cell line after 24 hours of treatment at 30 and 40 *μ*g/ml dosages. The data were provided as SOD, CAT, GSH, and MDA enzyme activity and mean SD (*n* = 3). Statistical significance is indicated by ^*∗*^*p* < 0.05 and ^#^*p* < 0.001 in contrast to the “control” group.

## Data Availability

The corresponding author can provide all available data integrated into the manuscript.
